This article has been retracted.

# MicroRNA-1269 is downregulated in glioblastoma and its maturation is regulated by long non-coding RNA SLC16A1 Antisense RNA 1

**DOI:** 10.1080/21655979.2022.2070581

**Published:** 2022-05-24

**Authors:** Zhibin Jin, Heyang Li, Yinbo Long, Rong Liu, Xiaoguang Ni

**Affiliations:** a Department of Neurosurgery, Cangzhou Central Hospital, Cangzhou City, People’s Republic of China; b Traditional Chinese Medical Science Hall, Cangzhou Central Hospital, Cangzhou City, People’s Republic of China

**Keywords:** MiR-1269, SLC16A1-AS1, glioblastoma, proliferation, maturation

## Abstract

MicroRNA-1269 (miR-1296) promotes esophageal cancer. However, its role in other cancers, such as glioblastoma (GBM) is unclear. We predicted that miR-1269 might interact with long non-coding RNA (lncRNA) SLC16A1 Antisense RNA 1 (SLC16A1-AS1), a critical player in GBM. We then studied the interaction between SLC16A1-AS1 and miR-1269 in GBM. In this study, paired GBM and non-tumor tissues were used to analyze the expression of SLC16A1-AS1 and premature and mature miR-1269. The interaction of SLC16A1-AS1 with premature miR-1269 was analyzed with RNA pull-down assay and dual-luciferase reporter assay. Cellular fractionation assay was applied to determine the subcellular location of SLC16A1-AS1. Overexpression assays were applied to determine the role of SLC16A1-AS1 in miR-1269 maturation. BrdU, Transwell and cell apoptosis assays were performed to analyze the role of SLC16A1-AS1 and miR-1269 in GBM cell proliferation, migration, and invasion. Interestingly, we observed the upregulation of premature miR-1269 and downregulation of mature miR-1269 in GBM. SLC16A1-AS1 was also overexpressed in GBM. The direct interaction of SLC16A1-AS1 with premature miR-1269 was observed. SLC16A1-AS1 suppressed miR-1269 maturation and promoted cell proliferation, migration, and invasion, and inhibited cell apoptosis, while miR-1269 displayed the opposite trend. SLC16A1-AS1 partly reversed the effects of miR-1269 on GBM cell proliferation, movement and apoptosis. Moreover, SLC16A1-AS1 overexpression increased the level of ki-67, CDK4 and Bcl-2 in LN-229 and LN-18 cells. However, miR-1269 could partly reverse the effect of SLC16A-AS1 on protein levels. Overall, miR-1269 is downregulated in GBM and its maturation is regulated by SLC16A1-AS1.

## Highlights

- SLC16A1-AS1 was overexpressed in GBM;
- MiR-1269 maturation was inhibited in GBM;
- SLC16A1-AS1 suppresses miR-1269 maturation in GBM.

## Introduction

Glioblastoma (GBM) refers to Grade IV glioma, the most common type of brain tumor [1,2]. It is a highly aggressive brain cancer and grows fast. Although GBM rarely spreads to distant organs, it can invade nearby brain tissues, leading to a high mortality rate [3]. In general, patients with GBM can only survive 12 to 18 months after initial diagnosis, with a 5-year survival rate of as low as 5% [4,5]. Although GBM patients can be treated with surgical resection with increased survival time, there is no cure for GBM [6]. Even worse, with population aging and environmental pollution aggregating, the incidence of GBM is increasing in many countries [7]. Therefore, novel therapies are needed.

Although lacking protein-coding capacity, microRNAs (miRNAs) with approximately 20 nucleotides in length [8] and long non-coding RNAs (lncRNAs) affect protein synthesis [9,10] to regulate cancer development, suggesting their potential role as targets for targeted therapy. Accumulating evidence has shown that dysregulation of miRNAs and lncRNAs are involved in many human cancers, including GBM [11,12]. For instance, Yan et al. reported that lncRNA ADAMTS9-AS2 blockage inhibits GBM progression via regulating the FUS/MDM2 ubiquitination axis [13]. Liao et al. demonstrated that lncRNA MALAT1 facilitates the malignancy of GBM via the miR-199a/ZHX1 axis [14]. Shou et al. revealed that lncRNA HOXA-AS2 is upregulated in GBM and promotes cancer development via regulating the miR-885-5p/RBBP4 axis [15]. MiR-34a expression is downregulated in GBM tissues and inhibits GBM progression [16]. A recent study showed that lncRNA SLC16A1 Antisense RNA 1 (SLC16A1-AS1, 1522 nt, chromosome 1) downregulates miR-149 through methylation to promote GBM cell proliferation [17]. However, the role of SLC16A1-AS1 in GBM remains to be further analyzed. We predicted that lncRNA SLC16A1-AS1 might bind to premature miR-1269 (22 nt, chromosome 4), a previously characterized oncogenic miRNA [18], to affect its maturation, thereby affecting GBM progression, and analyzed the interaction between SLC16A1-AS1 and miR-1269 in GBM.

## Materials and methods

### Patients and clinical samples

GBM and adjacent non-tumor tissues were donated by 50 patients who were admitted to Cangzhou Central Hospital between June 2020 and June 2021 after approval by the Ethics Committee of Cangzhou Central Hospital. Patients were included if they 1) were diagnosed as GBM through histopathological analysis; 2) not treated with therapies toward GBM, such as surgical resection, chemotherapy or radiation therapy prior to admission; 3) received surgical resection of the primary tumors after admission. Patients were excluded if they had 1) mental disorders and 2) infectious diseases. After surgical resection, both GBM and non-tumor tissues were obtained by dissection and stored in liquid nitrogen. All participants signed informed consent. All procedures were approved by the Ethics Committee of Cangzhou Central Hospital and operated in keeping with the standards set out in the Announcement of Helsinki and laboratory guidelines of research in China. Table 1 shows the patients’ clinical data.

**Table 1.** Associations between SLC16A1-AS1 and mature miR-1269 expression and patients’ clinical data

Parameter	Total	SLC16A1-AS1		P	Mature miR-1269		P
		Low	High		Low	High	
Age (years)							
<50	18	10	8	>0.05	7	11	>0.05
≥50	32	15	17		18	14	
Gender							
Female	20	8	12	>0.05	13	7	>0.05
Male	30	17	13		12	18	
Tumor size							
<3 cm	22	17	5	0.0006	4	18	0.00006
≥3 cm	28	8	20		21	7	
Necrosis							
Yes	10	4	6	>0.05	6	4	>0.05
No	40	21	19		19	21	
IDH mutation	5	2	3	>0.05	3	2	>0.05
H3K27 mutation	19	9	10	>0.05	10	9	>0.05
WHO grade							
I–II	24	12	12	>0.05	13	11	>0.05
III–IV	26	12	14		14	12	

### Cells and transfections

LN-229 and LN-18 human GBM cell lines (ATCC, USA) were cultured in DMEM/F12 medium 37°C in an incubator with 5% CO_2_ and 95% humidity. SLC16A1-AS1 (Accession: NR_103743.1) vector (pcDNA3.1) and miR-1269 (Accession: NR_031673.1) mimic were prepared by GenePharma. Overexpression of SLC16A1-AS1 and miR-1269 was achieved by transfecting SLC16A1-AS1 expression vector or miR-1269 mimic into cells using Lipofectamine 2000 reagent (Invitrogen) and confirmed 48 h later by RT-qPCR.

### Total RNA isolation

Total RNAs were extracted from about 10^7^ *in vitro* cultured cells or 0.03 g paired tissue samples using Aurum total RNA mini kit (Bio-Rad) and eluted in RNase-free water. Their concentration and integrity were analyzed using 2100 Bioanalyzer (Agilent). RNA samples with concentration > 1000 ng/µl and RIN value higher than 9.0 were used in subsequent analyses.

### Preparation of cDNA samples and RT-qPCR

Synthesis of cDNA was done through reverse transcription (RT) using PrimeScript RT-PCR Kit (Takara). After that, 1 µl cDNA sample was used as the template to perform qPCR on StepOne™ Real-Time PCR System (Thermo Fisher Scientific) to determine the expression of miR-1269 and SLC16A1-AS1 with U6 and 18S rRNA as internal controls, respectively. Ct value normalizations were performed with the 2^−ΔΔCt^ method[19]. Primer sequences were TGGATTGCCTAGACCAGGG and GCTGGAGACCAGGGAAGCC for premature miR-1269; CTGGACTGAGCCGTGCTAC and poly(T) for mature miR-1269; CTCGCTTCGGCAGCACAT and AACGATTCACGAATTTGCG for U6; TGGACGATGCATATGTGGG and CACGTTGGTTATGCGGTCA for SLC16A1-AS1; and GTAACCCGTTGAACCCCAT and CCATCCAATCGGTAGTAGC for 18S rRNA.

### Cellular fraction preparation and gene expression analysis

Both nuclear and cytoplasm fractions were prepared from 10^7^ cells using the Nuclear/Cytosol Fractionation Kit (Cat# K6911, Cell Biologics Inc.). In brief, cells were washed with ice-cold PBS, lysed on ice, and centrifuged at 1200 g for 20 min. The supernatant was collected as cytoplasm sample. The pellets were further subjected to nuclear lysis to prepare nuclear lysate. RNAs were isolated from both fractions and subjected to RT-PCR using QIAGEN OneStep RT-PCR Kit (QIANGEN, Shanghai, China) on ProFlex™ 2 x 384-well PCR System (Thermo Fisher Scientific) to detect SLC16A1-AS1 expression. PCR products were analyzed on agarose gels, stained with ethidium bromide, and analyzed using the method of delta Ct to determine the expression of target genes.

### RNA-RNA pulldown assay

Transcripts of SLC16A1-AS1 wild-type (SLC16A1-AS1-WT), SLC16A1-AS1 mutant (SLC16A1-AS1-mut) and a negative control (NC) were obtained through *in vitro* transcription, purified using MEGAclear™ Transcription Clean-Up Kit and labeled with biotin at 3’ end using Life Technologies Biotin 3’ End DNA Labeling Kit. The two labeled RNA samples, Bio-NC and Bio-SLC16A1-AS1, were transfected into cells, and cells were lyzed 48 h later. RNA–RNA complexes were pulled down using Pierce™ Streptavidin Magnetic Beads (Thermo Fisher Scientific) and eluted using elution buffer from the beads on DynaMag™-96 Side Magnet (Thermo Fisher Scientific). MiR-1269 in the complex was determined using RT-qPCR.

### Dual luciferase reporter assay

Dual-luciferase assay was performed using Dual-Luciferase® Reporter Assay System (Promega). Briefly, luciferase reporter vectors of NC (no binding site of premature miR-129), SLC16A1-AS1-WT and SLC16A1-AS1-mut were constructed using pGL3 Luciferase Reporter Vector (Promega Corporation) as the backbone. Cells were transfected with premature miR-1269, NC vector (NC group), SLC16A1-AS1-WT or SLC16A1-AS1-mut, and luciferase activity was determined 48 h later.

### Cell BrdU incorporation assay

Cell proliferation was analyzed by directly measuring DNA synthesis using BrdU incorporation assay [20] with BrdU Cell Proliferation ELISA Kit (ab126556, Abcam). Briefly, cells were harvested at 48 h post-transfections, washed with PBS, and incubated in fresh medium supplemented with BrdU (10 μM) for 2 h. Cells were then fixed after three times PBS wash and incubated with anti-BrdU-antibody (peroxidase-coupled, Sigma-Aldrich) for 2 h. After that, cells were further incubated peroxidase substrate tetramethylbenzidine for 1 h, and OD values at 450 nm were determined using BioTek Synergy HTX Multimode Reader (Agilent BioTek). Cell proliferation was calculated and normalized by setting OD values at 450 nm of the control group to value ‘1’.

### Cell apoptosis assay

Cell apoptosis assay was determined using a FITC Annexin V Apoptosis Detection Kit (BD Biosciences, USA). Briefly, cells were harvested and incubated with PI and FITC annexin V solution for 15 min and subjected to BD LSR II flow cytometry to analyze cells apoptosis (BD Biosciences, USA).

### Transwell assay

Transwell assays were used to analyze cell migration and invasion abilities. For invasion assay, Transwell chambers were pre-coated with 0.5 mg/ml Matrigel. Cells were collected at 48 h post-transfection, resuspended in serum-free medium and loaded to the upper chambers with 10^5^ cells per chamber. Cell movement was induced by 20% FBS in the lower chamber for 24 h. After stained with 0.1% crystal violet, cells were observed and counted under an Olympus CX33 modern trinocular microscope.

### Western blot

Total proteins were extracted by Radioimmunoprecipitation assay (RIPA) kit (Beyotime, Beijing, China) and the bicinchoninic acid (BCA) kit (Beyotime) was performed to detect the protein concentration. The protein was divided by PAGE and transferred to specific membranes (Millipore). Subsequently, the membranes were maintained with 5% skimmed milk for 1 h and incubated overnight at 4°C with specifc primary, including Bcl-2 (1:1000, ab32124, Abcam), CDK4 (1: 2000, ab137675, Abcam), Ki-67 (1:1000, ab205718, Abcam), GAPDH (1: 2000, ab9845, Abcam). were incubated overnight with the membranes at 4°C. Then, the membranes were incubated with the secondary antibodies for 1 h and then quantified by the ECL detecting system (Thermo Scientific, USA). GAPDH was used as the loading control. Finally, Quantity One version 4.2.1 (Bio-Rad Laboratories, Inc.) was utilized to analyze the separated proteins.

### Statistical analysis

All data were expressed as mean ± standard deviation (SD) of three biological replicates and compared. Differences between paired tissue samples were analyzed with paired t test and among more than 2 independent groups were explored with ANOVA Tukey’s test. Patients were divided into high and low SLC16A1-AS1 or miR-1269 level groups with the cutoff value being the median SLC16A1-AS1 or miR-1269 level in GBM tissue. Associations between patients’ clinical data and SLC16A1-AS1 levels in GBM tissues were analyzed with chi-squared test. A p < 0.01 was considered statistically significant.

## Results

### Differential expression of SLC16A1-AS1 and miR-1269 in GBM

We predicted that SLC16A1-AS1 and premature miR-1269 might interact with each other (shown below). Therefore, SLC16A1-AS1 may participate in miR-1269 maturation. To test this possibility, differential expressions of SLC16A1-AS1 and miR-1269 (mature and premature) in GBM were analyzed using RT-qPCR. It was observed that SLC16A1-AS1 (Figure 1a, p < 0.01) and premature miR-1269 (Figure 1b, p < 0.01) were upregulated in GBM tissues (n = 50) compared to paired non-tumor tissues (n = 50). In contrast, mature miR-1269 was downregulated in GBM tissues (n = 50) compared to non-tumor tissues (n = 50) (Figure 1c, p < 0.01). It is worth noting that SLC16A1-AS1 and miR-1269 (mature) expression levels were not significantly different among patients with different tumor grades. Among the 50 patients included in this study, IDH and H3K27 mutations were found in 5 and 19 cases, respectively. No close association between IDH and H3K27 mutations and SLC16A1-AS1 and miR-1269 (mature) expression levels were observed. Therefore, increased SLC16A1-AS1 expression and inhibited miR-1269 maturation may participate in GBM.

**Figure 1.** Differential expression of SLC16A1-AS1 and miR-1269 in GBM. After RNA isolation, differential expression of SLC16A1-AS1 (a), premature miR-1269 (b), and mature miR-1269 (c) in GBM (n = 50) and paired non-tumor tissues (n = 50) were analyzed using RT-qPCR. ** p < 0.01.

### Associations between SLC16A1-AS1 and mature miR-1269 expression and patients’ clinical data

To explore the potential role of SLC16A1-AS1 and miR-1269 in GBM, associations between patients’ clinical data and SLC16A1-AS1 levels in GBM tissues were analyzed with chi-squared test. As shown in Table 1, SLC16A1-AS1 and miR-1269 levels were closely correlated with tumor size, but not other clinical data (Necrosis), suggesting the involvement of SLC16A1-AS1 and miR-1269 in GBM.

### Correlations between SLC16A1-AS1 and mature or premature miR-1269 levels

Since SLC16A1-AS1 was predicted to bind to premature miR-1269, the correlation of SLC16A1-AS1 with mature or premature miR-1269 was analyzed with Pearson’s correlation coefficient. It was observed that SLC16A1-AS1 was significantly and positively correlated with premature miR-1269 (Figure 2a). In contrast, SLC16A1-AS1 and mature miR-1269 were inversely and significantly correlated (Figure 2b), supporting the involvement of SLC16A1-AS1 in miR-1269 maturation.

**Figure 2.** Correlations between SLC16A1-AS1 and mature or premature miR-1269. The correlation of SLC16A1-AS1 with mature (a) or premature miR-1269 (b) was analyzed using Pearson’s correlation coefficient.

### Binding of premature miR-1269 to SLC16A1-AS1

To test the possible involvement of SLC16A1-AS1 in miR-1269 the maturation, subcellular SLC16A1-AS1 location in LN-229 and LN-18 cells were analyzed. It was observed that SLC16A1-AS1 could be detected in both nuclear and cytoplasm fractions of these cells (Figure 3a). Prediction of the binding of premature miR-1269 to SLC16A1-AS1 using IntaRNA 2.0 revealed potential base pairing between them (Figure 3b). SLC16A1-AS1 mutant (SLC16A1-AS1-mut) was designed (indicated by red letters in Figure 3b). The direct interaction between SLC16A1-AS1 wild-type (SLC16A1-AS1-WT) and SLC16A1-AS1-mut and premature miR-1269 was confirmed by RNA–RNA pulldown assay and dual-luciferase reporter assay. RNA–RNA pulldown revealed increased premature miR-1269 accumulation in bio-SLC16A1-AS1-WT group, but not bio-SLC16A1-AS1-mut group, suggesting the direct interaction between them (Figure 3c, p < 0.01). Dual-luciferase reporter assay showed that compared to NC group, premature miR-1269 reduced the luciferase activity of bio-SLC16A1-AS1-WT vector, but not bio-SLC16A1-AS1-mut vector, further confirming the direct interaction between them (Figure 3d, p < 0.01).

**Figure 3.** Subcellular location of SLC16A1-AS1 in GBM cells and the direct interaction between SLC16A1-AS1 and premature miR-1269. Subcellular location of SLC16A1-AS1 (a) in LN-229 and LN-18 cells. SLC16A1-AS1 mutant (SLC16A1-AS1-mut) was designed (indicated by red letters in Figure 3b). The direct interactions between SLC16A1-AS1 wild-type (SLC16A1-AS1-WT) and SLC16A1-AS1-mut and premature miR-1269 were confirmed by RNA-RNA pulldown assay (b) and dual luciferase reporter assay (c). ** p < 0.01.

### SLC16A1-AS1 regulates miR-1269 maturation

To test the role of SLC16A1-AS1 in miR-1269 maturation, LN-229 and LN-18 cells were overexpressed with SLC16A1-AS1 or miR-1269 (Figure 4a, p < 0.01). SLC16A1-AS1 decreased mature miR-1269 accumulation (Figure 4b, p < 0.05), but increased premature miR-1269 accumulation (Figure 4c, p < 0.01). Therefore, SLC16A1-AS1 may suppress miR-1269 maturation in GBM cells.

**Figure 4.** SLC16A1-AS1 regulates the maturation of miR-1269. SLC16A1-AS1 or miR-1269 were overexpressed in LN-229 and LN-18 cells to further explore the interaction between them. Overexpression was confirmed every 24 h until 96 h (a). The role of SLC16A1-AS1 in regulating the expression of mature (b) and premature (c) miR-1269 was analyzed using RT-qPCR. ** p < 0.01.

### Roles of SLC16A1-AS1 and miR-1269 in GBM cell behaviors

BrdU, Transwell and apoptosis assays were performed to explore the roles of SLC16A1-AS1 and miR-1269 in regulating GBM cell behaviors. SLC16A1-AS1 increased cell proliferation, migration, and invasion, while miR-1269 showed opposite effects (p < 0.01). SLC16A1-AS1 also suppressed the inhibitory effects of miR-1269 on GBM cell proliferation, migration, and invasion (Figure 5a-c, p < 0.01). Moreover, SLC16A1-AS1 significantly inhibited and miR-1269 promoted GBM cell apoptosis. The promotion effect of miR-1269 on apoptosis of GBM cells was reversed by upregulating SLC16A1-AS1 expression (Figure 5d, p < 0.01). Therefore, SLC16A1-AS1 may regulate GBM cell proliferation, invasion, migration, and apoptosis through miR-1269. The representative images of migration, invasion, and apoptosis assays were presented in Supplemental Figure 1, 2 and 3, respectively. Western blot was conducted to explore protein levels of relative genes in proliferation (Ki-67), cell cycle (CDK4) and apoptosis (Bcl-2). As revealed in Figure 5e (p < 0.01), SLC16A1-AS1 overexpression upregulated and miR-1269 inhibited the level of ki-67, CDK4 and Bcl-2 in LN-229 and LN-18 cells. The stimulation effects of SLC16A1-AS1-induced on proteins level was partially rescued by miR-1269.

**Figure 5.** Effects of SLC16A1-AS1 and miR-1269 on GBM behaviors. BrdU and Transwell assays were performed to measure GBM cell proliferation (a), migration (b), and invasion (c). Cell apoptosis assay was performed to detect the apoptosis of (c) LN-229 and (d) LN-18 cells. Western blot was performed to detect protein levels of ki-67, CDK4 and Bcl-2 (e).** p < 0.01.

## Discussion

This study analyzed the differential expression of miR-1269 and SLC16A1-AS1 in GBM and their interactions in GBM. The results revealed the increased SLC16A1-AS1 expression and inhibited miR-1269 maturation in GBM. Most importantly, our study showed that miR-1269 maturation in GBM cells is likely regulated by SLC16A1-AS1.

The role of SLC16A1-AS1 has been studied in several types of cancers, such as liver cancer and GBM [17,18]. However, it plays opposite roles in the progression of different cancers. Pei et al. reported that SLC16A1-AS1 is downregulated in hepatocellular carcinoma and inhibits multiple-cell behaviors, such as migration and invasion by regulating the miR-301b-3p/CHD5 axis so as to suppress cancer progression and increase cancer cell sensitivity to radiosensitivity [19][21]. In contrast, SLC16A1-AS1 is upregulated in GBM and regulates miR-149 methylation to promote cell proliferation [17]. We found that SLC16A1-AS1 is upregulated in GBM tissues. SLC16A1-AS1 overexpression promotes GBM cell proliferation and movement and suppresses GBM cell apoptosis. Overexpression of SLC16A1-AS1 enhanced the expression of ki-67 and CDK4 and Bcl-2 in LN-229 and LN-18 cells, while the stimulating effect of SLC16A1-AS1-induced on protein levels was neutralized by miR-1269. In addition, SLC16A1-AS1 expression is only correlated with patients’ tumor size, but not other clinical factors. Therefore, SLC16A1-AS1 may mainly regulate tumor growth to promote GBM progression. However, this study only explored the effects of SLC16A1-AS1 overexpression, but not SLC16A1-AS1 knockdown, which is technically challenging. The role of SLC16A1-AS1 in GBM should be further analyzed by knockdown experiments.

Previous studies have extensively reported the oncogenic role of miR-1269 in cancers [18,22,23]. For instance, miR-1269 is upregulated in esophageal cancer and predicts patients’ poor survival [18]. MiR-1269 targets TGF-β1 to promote osteosarcoma [22]. MicR-1269 overexpression targets RASSF9 to regulate AKT, thereby promoting gastric cancer progression [23]. However, its expression pattern and function in GBM are unclear. Interestingly, we observed miR-1269 downregulation in GBM. miR-1269 overexpression inhibits GBM cell proliferation, migration, and invasion and promotes GBM cell apoptosis. Therefore, like SLC16A1-AS1, miR-1269 may have opposite roles in different cancers.

SLC16A1-AS1 is detected in both nuclear and cytoplasm fractions of GBM cells. Interestingly, SLC16A1-AS1 directly interacts with premature miR-1269, and SLC16A1-AS1 overexpression in GBM cells suppresses miR-1269 maturation. To produce mature miRNAs, premature miRNAs should be transported from the nucleus to the cytoplasm [24]. Therefore, SLC16A1-AS1 in the nuclear fraction may sponge premature miR-1269 to suppress their movement and maturation. Our study is the first to report the regulation of miR-1269 maturation by a lncRNA.

## Conclusion

SLC16A1-AS1 is overexpressed in GBM. SLC16A1-AS1 in the nuclear fraction may sponges premature miR-1269, thereby suppressing its maturation to promote cancer cell proliferation. With the increased understanding of the role of lncRNAs in GBM [25], lncRNAs are expected to serve as potential targets to treat GBM.

## Supplementary Material

Supplemental Material

## Data Availability

The data that support the findings of this study are available on request from the corresponding author.
